# Inverse Kinematics of Concentric Tube Robots in the Presence of Environmental Constraints

**DOI:** 10.1155/2021/4107732

**Published:** 2021-08-14

**Authors:** Mohammad Jabari, Manizhe Zakeri, Farrokh Janabi-Sharifi, Somayeh Norouzi-Ghazbi

**Affiliations:** ^1^Faculty of Mechanical Engineering, University of Tabriz, Tabriz, Iran; ^2^Department of Mechanical and Industrial Engineering, Ryerson University, Toronto, ON, Canada M5B 2K3; ^3^Department of Biomedical Engineering, Ryerson University, Toronto, Canada

## Abstract

Inverse kinematics (IK) of concentric tube continuum robots (CTRs) is associated with two main problems. First, the robot model (e.g., the relationship between the configuration space parameters and the robot end-effector) is not linear. Second, multiple solutions for the IK are available. This paper presents a general approach to solve the IK of CTRs in the presence of constrained environments. It is assumed that the distal tube of the CTR is inserted into a cavity while its proximal end is placed inside a tube resembling the vessel enabling the entry to the organ cavity. The robot-tissue interaction at the beginning of the organ-cavity imposed displacement and force constraints to the IK problem to secure a safe interaction between the robot and tissue. The IK in CTRs has been carried out by treating the problem as an optimization problem. To find the optimized IK of the CTR, the cost function is defined to be the minimization of input force into the body cavity and the occupied area by the robot shaft body. The optimization results show that CTRs can keep the safe force range in interaction with tissue for the specified trajectories of the distal tube. Various simulation scenarios are conducted to validate the approach. Using the IK obtained from the presented approach, the tracking accuracy is achieved as 0.01 mm which is acceptable for the application.

## 1. Introduction

Nowadays, continuum robots (CRs) have found widespread applications in medicine, especially in minimally invasive surgeries (MIS). Catheters are an example of CRs that are widely used in MIS. In recent years, comprehensive researches have been done on the design, manufacturing, and development of steerable catheters.

CRs could be modeled using two main approaches: (i) Cosserat rod theory and (ii) constant curvature [1–4]. The former provides a precise model of CRs using differential equations [5–7] while the latter provides a simpler model with less time-cost and still acceptable accuracy [8, 9]. Lyons et al. [10] presented a new method of optimization in IK for medical devices to plan configurations with anatomically constrained for reaching specified targets. In this paper, they calculate start position and orientation and a geometric representation of the physical environment extracted from preprocedure medical images. Forward and inverse kinematics of concentric tube continuum robots (CTCRs) using various geometrical approach are investigated in [11, 12], respectively. Anor et al. [13] presented a novel systematic approach to optimize the design of CTCRs for neurosurgical procedures. These procedures require that the robot approach specified target areas while navigating and operating within an anatomically constrained workspace. A particular advantage of this approach is that it identifies the need for either fixed-curvature versus variable-curvature sections. Due to the vast variety of applications in concentric tube robots, the optimization of concentric tube robots has always been alluring for researchers. For example, a new design of CTCR which is well suited to MIS inside small body cavities such as the heart is presented in [14]. This paper presents a generalized pattern search to optimize concentric tube robots while they can reach the target point with minimal curvature and length. Runge et al. [15] used evolutionary algorithms such as genetic algorithm to optimize a soft robot. Bodily et al. [16] used a genetic algorithm to optimize the reachability, dexterity, and manipulability of a multisegment continuum robot. Luo et al. [17] designed a concentric tube manipulator that is appropriate for surgical environments. They presented a new topology of the tubes for the concentric tube robot, which can increase the stable workspace because it allows the usage of larger tube curvatures and/or curve lengths. Davarpanah et al. [18] optimized a concentric tube robot using a genetic algorithm which allows them to reach the specific destination with high accuracy. Lloyd et al. [19] presented a novel model for optimizing a task-specific in millimeter-scale for magnetically actuated soft continuum robots used in medical applications. Finally, most similar to our work, Cheong et al. [20] applied a computational method to find optimal designs of continuum robots while considering reachability constraints.

This paper contributes to the field by finding an optimized inverse kinematic solution for a three-segment CTCR so that for a given position, the robot configuration would occupy minimized space. The proposed algorithm is very beneficial in MIS, where the robot needs to work in a tight space. Moreover, the optimized solution meets a safety interaction criterion at the base of the CR. In practice, when the robot inserts to an organ cavity, its shaft body would remain in the colons or vessels connected to that cavity. So, it is important that at the base of the robot, which is inside a tighter space, the CR does not apply forces to the surrounding tissues that may hurt.

In MIS applications, the robot is ideally expected to perform its mission with occupying the least possible workspace. To address this issue, in this paper, an algorithm is proposed that helps the minimum number of segments of a three-segment CR be involved in achieving a target point. Moreover, the robot-environment contact is modeled in the form of a spring which allows to apply interaction-force/displacement constraints to the base of the robot which assures a safe interaction. Finally, the research is concluded in Section 4.

## 2. Forward and Inverse Kinematics

In this section, the structure of the constant and variable length of a three-segment CTCR is described. The modeling assumptions of the CR are summarized as follows.

- The bending motion of the robot is planar
- The curvature of the robot backbone is supposed to be constant
- The curvature of each segment of the robot remains constant, thus, the central backbone is always located within a plane

Figure 1 shows a three-segment concentric tube continuum robot. Based on the following assumption, the constant curvature approach is utilized to model the system.

The parameters used to describe the model of a three-segment continuum robot are listed in Table 1.

Equation (1) calculates the length change of each segment.

(1) $$\begin{array}{c} L_{i}=L_{i0}+\Delta L_{i}, \end{array}$$

where *L*_*i*0_ is the length of the *i*^th^ segment in the primary situation of insertion, and Δ*L*_*i*_ is the decrease or increase in the *i*^th^ segment length which is task-dependent. Then, Eq. (2) shows the total length of the catheter.

(2) $$\begin{array}{c} L=\overset{n}{\underset{i=1}{\sum }}L_{i}=\overset{n}{\underset{i=1}{\sum }}\left(L_{\text{i}0}+\Delta L_{i}\right), \end{array}$$

### 2.1. Coordinate Systems

Figure 2 presents the relations between actuator space, configuration space, and task space. The actuator space includes tube lengths, the configuration space covers the robot bending angles and the insertion length, and finally, the task space is relevant to the end effector's position and orientation.

The coordinate systems for a single-segment continuum robot (see Figure 3) are described as follows.

1. *Base Coordinate System*. The base coordinate system represented by {*b*} = {*x*, *y*, *z*}
2. *End Coordinate System*. The coordinate system is located at the end point of the tube (i.e., the intersection of the tube with its nearby tube). The coordinate system is shown by *E*_*i*_ = {*x*_*i*_, *y*_*i*_, *z*_*i*_}, *i* = 1, 2, 3 for a three-segment catheter

### 2.2. Kinematics of Multisegment Robot

For the slender bar model, the curvature is not a constant and it can be widely used [21, 22]. As mentioned previously, the constant curvature approach is used to model the kinematics of the robot (Figure 3) [23, 24].

The general mapping between the task space and the configuration space can be obtained by a homogeneous transformation matrix (Eq. (3)),

(3) $$\begin{array}{c} T=\left[\begin{array}{cc} R_{ot} & p\\ 0 & 1 \end{array}\right]=\left[\begin{array}{cc} \begin{array}{cc} c^{2}\varphi \left(c\left(kl\right)-1\right)+1 & -s\varphi c\varphi \left(c\left(kl\right)-1\right)\\ s\varphi c\varphi \left(c\left(kl\right)-1\right) & c^{2}\varphi \left(1-c\left(kl\right)\right)+c\left(kl\right) \end{array} & \begin{array}{cc} c\varphi s\left(kl\right) & \frac{c\varphi \left(1-c\left(kl\right)\right)}{k}\\ s\varphi s\left(kl\right) & \frac{s\varphi \left(1-c\left(kl\right)\right)}{k} \end{array}\\ \begin{array}{cc} -c\varphi s\left(kl\right) & -s\varphi s\left(kl\right)\\ 0 & 0 \end{array} & \begin{array}{cc} c\left(kl\right) & \frac{s\left(kl\right)}{k}\\ 0 & 1 \end{array} \end{array}\right], \end{array}$$

where *R*_*ot*_ represents the orientation of the end effector, *p* is the end position of the robot [25], *c* and *s* stand for cos and sin, respectively. Using the length and radius of the robot curvature shown in Figure 3, the angle  *α* can be calculated using

(4) $$\begin{array}{c} \alpha =\frac{l}{R}=kl, \end{array}$$

where *R*,  *l*, and *k* are the arc length, bending radius, and curvature, respectively. More details on how to obtain Eqs. (3) and (4) could be found in [25, 26]. The forward kinematic model of the three-segment CR can be obtained using

(5)  3bT= 0bT  10T  21T  32T.

### 2.3. Inverse Kinematic for a Multisegment Robot

Increased degrees of freedom (DOF) bring more redundancy for the robot configuration. As a result, there are no closed-form solutions for the multisegment robot inverse kinematic. Moreover, there would be multiple solutions for the problem of finding the inverse kinematics. To obtain the forward kinematic model, two different cases need to be considered for the bending angle of the distal segment [27] including *θ*_dist_ < 90° and 90° ≤ *θ*_dist_ ≤ 180°. The position of the central backbone of the catheter in the second and third segments is achieved using

(6) $$\begin{array}{c} \begin{array}{c} {\tilde{p}}_{2}=R_{ot}{\left(\alpha_{\text{prox}}\right)}^{-1}\left(p_{2}-p_{1}\right),\\ {\hat{p}}_{3}=R_{ot}{\left(\alpha_{\text{med}}\right)}^{-1}\left(\left(p_{3}-p_{1}\right)R_{ot}{\left(\alpha_{\text{prox}}\right)}^{-1}-p_{2}\right), \end{array} \end{array}$$

where the points *P*_0_^*T*^ = [*x*_0_ *y*_0_ *z*_0_], *P*_1_^*T*^ = [*x*_1_ *y*_1_ *z*_1_], *P*_2_^*T*^ = [*x*_2_ *y*_2_ *z*_2_], and *P*_3_^*T*^ = [*x*_3_ *y*_3_ *z*_3_] are the catheter base coordinate system, the intersection of the first and second segments, the intersection of the second and third segments, and the end-plate of the third segment, respectively. More details can be found in [27]. Vectors ${\tilde{p}}_{2}$ and ${\hat{p}}_{3}$ are local positions of the end-effector in the coordinate systems at the base of each tube.

### 2.4. Optimization Problem

The optimization problem is defined to minimize the tracking error between the catheter tip and the corresponding target position (*P*_ref_^*T*^ = [*x*_ref_ *y*_ref_ *z*_ref_]). Also, the optimized parameter would be the configuration parameters including bending and rotation angles and insertion length of each segment. According to the number of extended segments (e.g., when two or three tubes are inserted out from the overlapped tube), the catheter tip can be denoted by either ${\tilde{p}}_{2}$ or ${\hat{p}}_{3}.$ To form cost function, we first rearrange Eq. (6) as follows

(7) $$\begin{array}{c} \begin{array}{c} P_{2.\text{ref}}=P_{1}+R_{ot}\left(\alpha_{\text{prox}}\right){\tilde{p}}_{2}.\\ P_{3.\text{ref}}=P_{1}+R_{ot}\left(\alpha_{\text{prox}}\right)P_{2}+R_{ot}\left(\alpha_{\text{med}}\right)R_{ot}\left(\alpha_{\text{prox}}\right){\hat{P}}_{3}. \end{array} \end{array}$$

Next, the cost functions of the two-segment and three-segment catheter can be defined in the form of

(8) $$\begin{array}{c} J=\gamma {\left(p_{2.\text{ref}}-\left(p_{1}+R_{ot}\left(\alpha_{\text{prox}}\right){\tilde{p}}_{2}\right)\right)}^{T}\left(p_{2,\text{ref}}-\left(p_{1}+R_{ot}\left(\alpha_{\text{prox}}\right){\tilde{p}}_{2}\right)\right)+\alpha_{\text{prox}}^{2}+\alpha_{\text{dist}}^{2}, \end{array}$$

(9) $$\begin{array}{c} J=\gamma {\left(p_{3.\text{ref}}-\left(p_{1}+R_{ot}\left(\alpha_{\text{prox}}\right)p_{2}+R_{ot}\left(\alpha_{\text{med}}\right)R_{ot}\left(\alpha_{\text{prox}}\right){\overset{\wedge }{p}}_{3}\right)\right)}^{T}\left(p_{3.\text{ref}}-\left(p_{1}+R_{ot}\left(\alpha_{\text{prox}}\right)p_{2}+R_{ot}\left(\alpha_{\text{med}}\right)R_{ot}\left(\alpha_{\text{prox}}\right){\hat{p}}_{3}\right)\right)+\alpha_{\text{prox}}^{2}+\alpha_{\text{med}}^{2}+\alpha_{\text{dist}}^{2}, \end{array}$$

where *γ* is a weighting factor.

### 2.5. Safe Interaction Conditions

According to Figure 4, if you want the robot to be safely interacting with the texture, at first, the texture should be modeled into a spring, then, the amount of the allowed displacement for being in contact with the robot base should be obtained. Allowed ranges of the interaction force vary across surgical tasks. The size and fragility of the tissue are important parameters affecting the allowed force range.

In this paper, the following assumptions are made according to the literature [28, 29].

- Diameter of the main coronary arteries is about 4 mm [30]
- The maximum allowed force applicable to the texture is considered as 0.2 N. The texture stiffness, at the entrance of the cavity, is considered to be *k* = 100 N/m which corresponds to 2 mm displacement of the tissue which is acceptable (Eq. (10))

(10) $$\begin{array}{c} F=K\Delta x_{T}\Rightarrow \Delta x_{T}=\frac{F}{K}=\pm 2\text{ mm}. \end{array}$$

Δ*x*_*T*_ equals to the required displacement of *P*_*b*_ = (*x*, *y*, *z*) so that the catheter tip would reach to the target point.

(11) $$\begin{array}{c} \Delta x_{T}=\sqrt{{\left(x_{\text{new}}-x_{\text{old}}\right)}^{2}+{\left(y_{\text{new}}-y_{\text{old}}\right)}^{2}+{\left(z_{\text{new}}-z_{\text{old}}\right)}^{2}}, \end{array}$$

To obtain Δ*x*_*T*_, first, the shape of catheter corresponding to the desired tip catheter is obtained, and then among the multiple solutions, those solutions which are meeting the safety constraint at the point of *P*_*b*_ are accepted.

## 3. Results and Discussion

In this section, first, we simulated the kinematic model obtained in the previous section using MATLAB.

Figure 5 demonstrates the simulation results for the three-segment catheter. The robot configuration parameters corresponding to the target point of the catheter tip are listed in Table 2.

Figure 6 shows the mapping between the position of the robot end-effector and the configuration space variables. At each iteration, the bending and rotation angles change smoothly within [0 *π*] and [0 2*π*], respectively. Step-increment equals to 1.8° for *α* and 3.6° for *φ*. The number of the chosen sample points is 100. The weighting factor *γ* is set to 50.

### 3.1. Continuum Robot Workspace

In this section, the robot workspace for a single, two, and three-segment catheter is obtained and demonstrated. The variation range of the configuration parameters are shown in Table 3.

As illustrated in Figures 7–12, with the increase of the number of robot segments, the thickness of the clouds forming the workspace is increasing, which reflects an enlarged accessible space and increased precision of the three-segment catheter compared to single- or two-segment catheter. Hence, one can conclude that multisegment catheters are more appropriate choices for applications in which the catheter is supposed to operate in confined spaces.

### 3.2. Continuum Robot with Variable Length: Insertion Optimization

In this section, we consider a continuum robot with variable length. The purpose is to optimize the robot segment lengths while meeting the aforementioned constraints. The schematic of the proposed optimization algorithm is shown in Figure 13. In this diagram, first, concentric tube robot receives the desired point and then calculates the distance between the robot's tip and the desired point and increases the tube's length based on the calculations. If the desired point is in the range of tube 1, only segment 1 would be involved to help the end-effector reach the target point. Otherwise, the second and the third segments would be inserted to the workspace.

### 3.3. Optimization Example: A Catheter with Two Segments (No Insertion Is Allowed)

We consider a two-segment catheter of 120 mm length (60 mm for each segment). The target point is set to *P*^*T*^[−47.98  − 33.92 33.90]. Using the proposed algorithm, as it has been shown in Figures 14 and 15, after 2000 iterations, the optimal parameters of the robot including the bending and rotation angle of each segment can be observed in Tables 4 and 5.

According to Figure 14, the amount of the cost function after about 40 first iterations is approximately equal  *J* = 8.03.

We also consider the hypothetical target point in the coordinate system *P*^*T*^ = [40.85 77.24 26.97] of for the optimization of the three-segment catheter configuration space with a general length of 120 mm and a separate length of 40 mm for each segment.

As it can also be seen in Figure 15, the amount of the cost function, after about 60 first iterations, equals  *J* = 6.59.

The simulation results show that the catheter accuracy to approach the point in question is too much, also, a considerable amount of optimization, in the first several iterations, shows itself; as a result, it will be possible to reduce the iteration limit when the velocity of the process seems to be important to us.

### 3.4. Optimization Example: A Catheter with Two and Three Segments (Insertion Is Allowed)

As it was mentioned, in the variable-length catheter, considering the target point, first, the proximal segment length increases from its primary length considered to be zero to its final length, and this same trend for other links reports in order to approach the target point.

The three-segment catheter will have the same length for each segment which is 40 mm has been used, so as to simulate how to access the variable-length catheter.

We consider the target point at *P* = [34.85 17.11 62.22]^*T*^. After 2000 iterations, and after optimization using the genetic algorithm, and also using the cost function of Eq. (8), the amount of the shown response in the 2016 Matlab will be in the form of Table 6. According to these optimal parameters, the order of error is 0.01 mm for two segment catheter which is small in comparison to three segment catheter that has an error greater than 1 mm. Therefore, the variable-length catheter will use two-segment of its inner parts in order to approach the desirable point, and this same result has been shown in the last row of the first column. Also, the optimization amount of the two-segment cost function has been obtained to be the number of *J* = 1.1032 that is an appropriate amount for tracking the target point.

### 3.5. Optimization of the Three-Segment Catheter with Variable Length Having the Safe Interacting with Fragile Structures like Texture

We choose first the hypothetical point of *P* = [30.16 25.59 65.96]^*T*^ as the target point, for optimization of the three-segment catheter configuration space with variable length. In the simulations, we consider first the position of the robot tip at the entrance of the cavity in the form of the coordinate system of *B* = [0 0 10]^*T*^. At first, the optimization results for the point in question are shown in Table 7 without the safe interaction with the fragile structures like texture. If  *dB* < Δ*x*_*T*_, the obtained position and the parameters related to this position are correct, if not, another response is chosen.

According to these optimal parameters, the order of error is 0.01 mm for a two-segment catheter which is small in comparison to three segment catheter that has an error greater than  1 mm. Regarding the error amount, for each segment, the desirable link will be the second link. Also, the amount of the cost function for the two-segment of the variable-length catheter will be equal to 1.4539.

As you can see in Table 8, for the catheter safe interacting with fragile structures like texture, according to the Eqs. (8) and (9), at first, we obtained the safe limitation constraint for interacting with fragile structures like texture. Considering the two mentioned conditions, we take into consideration the maximum amount of the allowed force which is applied to the texture to be 0.2 N, and also the stiffness to be 100, at the entrance of the cavity. According to Eq. (10), the displacement amount at the contact point with the texture will be obtained as ±2 mm. Now, after required iterations from the population in the algorithm, in each of the robot segments, the correct link for approaching the chosen target point and the angle amounts of the catheter are obtained in the case that the distance amount of the robot is less than 2 mm.

According to the obtained error amount from the hypothetical target point and the tracked point in the three-segment catheter, it can be concluded that the three-segment catheter has an undesirable tracking for approaching the target point, and also according to the obtained points in the table second column, and the little error amount the catheter will use two segments from its inner parts for approaching to the desired point.

Also, the optimized cost function amount of the two-segment catheter is obtained to be 2.8294 which is an appropriate amount for tracking the target point. In the last row of the first column, the allowed displacement amount at the contact point with the texture has been gained which is equal to dB = 1.1641 mm, which is less than the indicated amount of 2 mm. This shows the catheter's safe interaction with the texture.

## 4. Conclusion

In this paper, the optimization and kinematic model of the continuum robot target tracking have been surveyed in two states of constant and variable lengths. To do this, the method of the constant curvature was applied, considering the bending of each segment of the robot in the Platform, extracting the forward kinematics for constant and variable lengths, and using inverse kinematics for the robot. This robot's being redundant has caused it not to require the closed-form solution for its inverse kinematic. For this reason, optimization and numerical solving methods have been used for tracking the target by the robot. Adding the possibility of the robot length change, the robot workspace and redundancy are increased, and we can use it to provide more dexterity. As it was done in this research, whereas the length changes of each one of the segments are influenced using the offered algorithm as a variable of the configuration space for approaching the target point, it is possible to use it as a tool for better control of the robot. Also, the robot movement limit will be more appropriate for environments like the vessels. In this paper, the results of the forward kinematics parts confirm the results of the inverse kinematics parts, and vice versa, which indicates the accuracy of the model. Also, for the part of the optimization of the multisegment catheter, the results also indicate the model appropriate accuracy in tracking the giving points for performing endovascular surgery. The average distal end positioning error is less than 1% for each segment of the catheter, which is an acceptable error for most real-time surgeries. In the final part, regarding force imposed onto the texture, and also the stiffness, the allowed distance amount with the texture causes the safe interaction. The implementation of the secure interaction with the texture and the trajectory results indicate the catheter has an accurate application in the medical procedure. Future works focusing on the addition of more constraints, and optimization of the distinguished constraints of the cost function, try to lessen the tracking errors and to improve the stability of the existing catheter. Also, tracking a certain path concerning the safe interaction with the texture for the catheter will be carried out.

## Figures and Tables

**Figure 1:** The scheme of a concentric tube robot comprising three precurved tubes.

**Figure 2:** Mapping between joint space variables, configuration space variables, and workspace variables.

**Figure 3:** The introduced parameters in the robot: (a) the geometric display of a robot segment and (b) the display from the above of the robot platform.

**Figure 4:** The safe interaction with the texture modeled by the spring.

**Figure 5:** Configuration of the three-segment catheter with bending and rotation angles.

**Figure 6:** Changes of the robot's final position according to the mapping of the configuration space variables.

**Figure 7:** One-segment catheter workspace in 2D.

**Figure 8:** One-segment catheter workspace in 3D.

**Figure 9:** Two-segment catheter workspace in 2D.

**Figure 10:** Two-segment catheter workspace in 3D.

**Figure 11:** Three-segment catheter workspace in 2D.

**Figure 12:** Three-segment catheter workspace in 3D.

**Figure 13:** Flow chart for finding an optimal inverse kinematics.

**Figure 14:** Genetic algorithm for best fitness target point in two-segment catheter.

**Figure 15:** Genetic algorithm for best fitness target point in three-segment catheter.

**Table 1:** The list of the nomenclatures used in this paper.

Symbol	Definition
*R*	The radius of curvature in the primary backbone is defined in the bending plate (the plate of *X*_1_*Z*_1_)
*α*	The bending angle in the primary backbone is defined in the bending plate (*X*_1_*Z*_1_ plate) at the point *O*′.
*φ* ∈ [0 2*π*]	The orientation angle of the robot which can rotate in the *xy* plate
*φ*_prox_, *α*_prox_	Rotation and bending angles of the first part of the catheter
*φ*_med_, *α*_med_	Rotation and bending angles of the second part of the catheter
*φ*_dist_, *α*_dist_	Rotation and bending angles of the third part of the catheter
*L*_0_	The primary length of the primary backbone
*A*_*i*_	The position of the *i*^th^ secondary backbone fixed in the lower platform
*B*_*i*_	The position of the *i*^th^ secondary backbone fixed in the upper platform
*O*	The center of the equilateral triangle made by the *A*_*i*_ points in the platform of {*x*, *y*, *z*}
*C*	The center of the equilateral triangle made by the *B*_*i*_ points in the platform of {*x*_1_, *y*_1_, *z*_1_}
*P* = [*x*_*c*_ *y*_*c*_ *z*_*c*_]^*T*^	The position vector stating the center coordinate of the upper platform of each segment according to the lower platform
*k*	Curvature
*v* = [*k* *φ*_*c*_ *l*]^*T*^	The configuration space vector
*n*	The number of robot segments
*R*_0*t*_ ∈ *R*^3×3^	The rotation matrix from the end disk coordinate system to the base coordinate system

**Table 2:** Three-segment continuum robot bending and rotation angles.

Angles	Segment 1	Segment 2	Segment 3
Bending angle (*α*)	63.24°	53.54°	35.58°
Rotation angle (*φ*)	49.80°	310.05°	178.89°
Length (mm)	73.26	36.63	76.21

**Table 3:** The simulation conditions for workspace.

Parameters	Single-segment	Two-segment	Three-segment
The length of each segment	120 mm	60 mm	40 mm
*α*_*i*_	[0 *π*]	[0 *π*/2]	[0 *π*/3]
*φ*_*i*_	[0 2*π*]	[0 2*π*]	[0 2*π*]

**Table 4:** Optimized results for reaching target point.

Section number	Optimal bending angle (degree)	Optimal rotation angle (degree)	Reaching point (mm)	Error (mm)
1	99.80	195.42	*X*: -40.81 *Y*: -33.64 *Z*: 33.73	*X*: 0.17 *Y*: 0.28 *Z*: 0.17
2	88.57	324.01		

**Table 5:** Optimized results for reaching target point.

Section number	Optimal bending angle (degree)	Optimal rotation angle (degree)	Reaching point (mm)	Error (mm)
1	98.34	53.36	*X*: 40.86 *Y*: 77.27 *Z*: 26.97	*X*: 0.01 *Y*: 0.03 *Z*: 0
2	99.33	151.98		
3	43.78	73.15		

**Table 6:** Optimized results for three-segment catheter with variable length.

Two-segment	Tracked point	Three-segment	Tracked point
*θ*_prox_ : 44.6093 *φ*_prox_ : 8.2412 *θ*_med_ : 38.9934 *φ*_med_ : 122.5938	*X*2: 34.837 *Y*2: 17.099 *Z*2: 66.199	*θ*_prox_ : 44.6093 *φ*_prox_ : 8.2412 *θ*_med_ : 38.9934 *φ*_med_ : 122.5938 *θ*_dist_ : 192.3173 *φ*_dist_ : 145.7034	*X*3: 17.4794 *Y*3: 32.5204 *Z*3: 61.4679
*J*: 1.1032 Link-num: 2			

**Table 7:** Optimized results for a three-segment catheter with variable length without interaction with fragile structures like texture.

Two-segment	Tracked point	Three-segment	Tracked point
*θ*_prox_ : 49.5561 *φ*_prox_ : 55.6513 *θ*_med_ : 41.6511 *φ*_med_ : 284.3094	*X*2: 30.1286 *Y*2: 25.5773 *Z*2: 65.9110	*θ*_prox_ : 53.3323 *φ*_prox_ : 49.0286 *θ*_med_ : 41.5474 *φ*_med_ : 255.1113 *θ*_dist_ : 124.2572 *φ*_dist_ : 284.6543	*X*3: 50.6561 *Y*3: 1.2243 *Z*3: 72.9058
*J*: 1.4539 Link-num: 2			

**Table 8:** Optimized results for three-segment catheter with variable length with interaction with fragile structures like texture.

Two-segment	Tracked point	Three-segment	Tracked point
*θ*_prox_ : 53.4391 *φ*_prox_ : 53.6859 *θ*_med_ : 47.2743 *φ*_med_ : 269.4255	*X*2: 30.0826 *Y*2: 25.5582 *Z*2: 65.8237	*θ*_prox_ : 53.4391 *φ*_prox_ : 53.6859 *θ*_med_ : 47.2743 *φ*_med_ : 269.4255 *θ*_dist_ : 299.592 *φ*_dist_ : 220.5672	*X*3: 24.9051 *Y*3: 22.4644 *Z*3: 61.0422
*J*: 2.8294 Link-num: 2 dB: 1.1641			

## Data Availability

The MATLAB code data used to support the findings of this study are available from the corresponding author upon request.
